The article "Curcumin Blunts IL-6 Dependent Endothelial‐to‐Mesenchymal Transition to Alleviate Renal Allograft Fibrosis Through Autophagy Activation" was retracted in 2021. Reasons: errors in the data; unreliable images; unreliable results or conclusions.

# Curcumin Blunts IL-6 Dependent Endothelial‐to‐Mesenchymal Transition to Alleviate Renal Allograft Fibrosis Through Autophagy Activation

**DOI:** 10.3389/fimmu.2021.656242

**Published:** 2021-05-28

**Authors:** Jiajun Zhou, Mengtian Yao, Minghui Zhu, Mengchao Li, Qiwei Ke, Bing Wu, Daming Wang

**Affiliations:** ^1^ Department of Emergency Intensive Care Unit, The Third Affiliated Hospital, Soochow University, Changzhou, China; ^2^ Department of Endocrine, Changzhou Hospital of Traditional Chinese Medicine, Changzhou, China

**Keywords:** endothelial‐to‐mesenchymal transition, allograft fibrosis, autophagy, curcumin, chronic allograft dysfunction

## Abstract

Fibrosis contributes to graft loss in chronic renal allograft injury. Endothelial‐to‐mesenchymal transition (EndMT) plays an important role in the development of fibrosis following kidney transplantation. Autophagy plays an important role in the homeostasis of diverse cell types including endothelial cells. Here we demonstrate that inhibition of autophagy by treatment with 3-methyladenine (3-MA) or by silencing autophagy-related (ATG)5 promoted interleukin (IL)-6–dependent EndMT in human umbilical vein endothelial cells (HUVECs) and human renal glomerular endothelial cells (HRGECs), and autophagy inactivation was associated with EndMT in patients with chronic allograft dysfunction. IL-6 level was significantly higher in the culture medium of HUVECs transfected with ATG5 siRNA or treated with 3-MA compared to the respective control groups. IL-6 application induced EndMT in HUVECs and HRGECs, whereas antibody-mediated neutralization of IL-6 suppressed EndMT induced by ATG5 silencing. The protective role of curcumin (Cur) against allograft fibrosis was confirmed in a rat kidney transplantation model of F344 donors to Lewis recipients. Curcumin—a natural polyphenol compound with known antifibrotic effects in various tissues—alleviated IL-6–induced EndMT and promoted autophagy in the allografted organ and in HUVECs. This is the first demonstration of the role of autophagy in renal allograft fibrosis; our findings indicate that curcumin can alleviate chronic renal allograft injury by suppressing IL-6–dependent EndMT *via* activation of autophagy.

## Introduction

Kidney transplantation is the most effective treatment for end-stage renal disease. Compared to dialysis, patients who undergo this procedure have a better quality or life and enhanced survival. However, the long-term survival rate of allograft recipients remains unsatisfactory. Chronic allograft dysfunction (CAD)—which is characterized by the progressive impairment of renal graft function—is the major cause of allograft loss (1, 2). CAD is a multifactorial process involving immunologic and nonimmunologic factors such as organ conservation, side effects of immunosuppressants, rejection, etc. (3) Given the complex causes of CAD, treatment options are limited. Allograft fibrosis, the main pathologic lesion of CAD, is caused by excessive extracellular matrix (ECM) production and abnormal deposition of fibrous connective tissue in the allograft (4). Myofibroblasts (MFBs), which produce ECM, are key players in this process (5).

The article "Curcumin Blunts IL-6 Dependent Endothelial‐to‐Mesenchymal Transition to Alleviate Renal Allograft Fibrosis Through Autophagy Activation" was retracted in 2021. Reasons: errors in the data; unreliable images; unreliable results or conclusions.

Most studies on renal fibrosis have focused on epithelial cells because of their abundance in kidney (accounting for 65% of all cells) (6, 7). Epithelial cells transform to myofibroblast through epithelial–mesenchymal transition (EMT) and play a critical role in occurrence of renal fibrosis. We previously showed that bortezomib alleviated renal allograft fibrosis by preventing tumor necrosis factor-α–induced EMT (8), although the underlying mechanism is unknown. Following kidney transplantation, many cell types including endothelial cells, bone marrow mesenchymal stem cells, and peripheral blood cells transform into MFBs to promote allograft fibrosis (9–11). Disruption of endothelial cell homeostasis contributes to the pathogenesis of the allografted organ (12). Endothelial‐to‐mesenchymal transition (EndMT) in endothelial dysfunction is another source of MFBs (13); in this process, endothelial cells downregulate vascular endothelial (VE)-cadherin, CD31 and CD34 and express mesenchymal cell markers including α-smooth muscle actin (α-SMA), collagen I and III, and fibronectin (FN).

Autophagy is an evolutionarily conserved cellular process involving the clearance of dysfunctional organelles, abnormal aggregated proteins and lipids, and pathogens that plays an important role in normal cell development, differentiation, and survival and tissue homeostasis (14, 15). The function of autophagy depends on specific organ and cell types. Dysregulation of autophagy has been reported in fibrotic diseases (16–18). Autophagy in endothelial cells is associated with diverse pathologic conditions. In human cardiac microvascular endothelial cells, defective autophagy promoted hypoxia-induced EndMT and induced myocardial fibrosis (19). In patients with type 2 diabetes, inadequate autophagy resulted in endothelial cell dysfunction (20); and loss of the autophagy-related (ATG)5 gene accelerated diabetic nephropathy and led to renal fibrosis (21). Conversely, enhancing autophagy prolonged cardiac transplant survival (22). And in a rat liver transplantation model, inhibiting autophagy had a protective effect on liver function (23). However, the role of endothelial cell autophagy in renal allografts is unclear.

The article "Curcumin Blunts IL-6 Dependent Endothelial‐to‐Mesenchymal Transition to Alleviate Renal Allograft Fibrosis Through Autophagy Activation" was retracted in 2021. Reasons: errors in the data; unreliable images; unreliable results or conclusions.

Immunosuppressants are widely used for the treatment of fibrosis, but nephrotoxicity is a side effect of some of these drugs and may cause fibrosis in the allografted organ. Additionally, current immunosuppressive schemes cannot prevent ECM deposition or promote ECM degradation. Curcumin, a natural polyphenol compound extracted from turmeric, has demonstrated antifibrotic effects in the heart, liver, and kidney (24–26). However, it has relatively low bioavailability and the peak plasma level does not reach the minimum effective concentration determined from *in vitro* studies (27). Curcumin was reported to block EMT in hepatocytes to alleviate hepatic fibrosis by promoting autophagy (28). Recent studies have shown that inactivation of autophagy in endothelial cells induces interleukin (IL)-6–dependent EndMT (29). In the present study, we investigated whether this contributes to the pathogenesis of CAD and examined the underlying mechanisms using human umbilical vein endothelial cells (HUVECs) and human renal glomerular endothelial cells (HRGECs). Additionally, we evaluated whether curcumin could alleviate IL-6–dependent EndMT by promoting autophagy *in vitro* and *in vivo* using a rat kidney transplantation model.

## Materials and Methods

### Reagents

Anti-CD31, Anti-α-SMA, Anti-IL-6 and Anti-VE-cadherin were purchased from Abcam (ab16669, ab7817, ab233706, ab33168, Abcam; Cambridge, UK). Autophagy related antibodies (Anti-Beclin1, Anti-LC3 I and II, Anti-P63, Anti-SQSTM1) and Anti-GAPDH antibodies were purchased from Cell Signaling Technology (4445,2524,8242, CST; Boston, USA). Anti-fibronectin antibodies were brought from Becton Dickinson and Company (610077, BD; New Jersey, USA). Anti-IL6 monoclonal IgG, control monoclonal IgG and Human recombinant IL-6 were purchased from Merck (I7901, I8765, HY-P7044, Merck; Darmstadt, Germany).3-MA and curcumin were purchased from Selleck chem (S2767, S1848, Selleck; Houston, USA). Myeloperoxidase (MPO) Activity Assay Kit was purchased from SIGMA (mak068, SIGMA; Saint Louis, USA). Superoxide dismutase (SOD) Activity Assay Kit was purchased from SIGMA (19160, SIGMA; Saint Louis, USA).

### Ethics Statement

The study protocol of transplant kidney biopsy or resection was in accordance with the ethical standards of the Declaration of Helsinki. The 2008 Declaration of Istanbul principles was strictly followed by us. We retrospectively included 22 kidney-transplanted patients in the third affiliated hospital of Soochow University who underwent a kidney graft biopsy or allograft resection from 2015-2020. The protocol of this study was approved by the local ethics committee of the third affiliated hospital of Soochow University. Informed written consent was given by the patients for the use of part of the tissues for scientific purposes.

The article "Curcumin Blunts IL-6 Dependent Endothelial‐to‐Mesenchymal Transition to Alleviate Renal Allograft Fibrosis Through Autophagy Activation" was retracted in 2021. Reasons: errors in the data; unreliable images; unreliable results or conclusions.

### Sample Collection

Total 22 allograft segments from patients, who received transplanted kidney nephrectomy or kidney biopsy from 2015-2020, were divided into two groups. Stable group (including 10 patients) was determined by their stable renal functions and no evidence of active rejection.12 patients were diagnosed with CAD according to their clinical symptoms and allograft pathological results. The demographics of patients in the CAD group and Stable group are given in **Table 1**.

**Table 1:** Patient demographics.

Clinical variables	CAD group	Stable group	P value
n	12	10	
Age (years, mean± S.D.)	35.13 ± 4.11	38.15 ± 2.81	NS
Men/Women	7/5	5/5	NS
BMI (kg/m^2^, mean ± S.D.)	21.11 ± 6.51	19.81 ± 7.81	NS
Transplant duration (years, range)	6.9(4.7-10.2)	5.7(3.1-9.4)	NS
Primary/secondary kidney transplant	12/0	10/0	NS
% PRA at transplant	0	0	NS
Immunosuppressive regimen			
Prednisone + MMF + Tac	6	5	
Prednisone + MMF + CsA	6	5	
Biochemical parameters			
Serum creatinine (μmol/l, mean ± S.D.)	309.1 ± 50.18	67.79 ± 15.13	<0.001
eGFR* (min/1.73 m^2^, mean ± S.D.)	20.1 ± 2.49	73.12 ± 4.98	<0.001

CAD, Chronic allograft dysfunction; BMI, body mass index; PRA, panel reaction antibody; MMF, mycophenolate mofetil; CsA, cyclosporine A; Tac, tacrolimus; eGFR, estimated glomerular filtration rate; S.D., standard deviation; NS, no significance. *eGFR was estimated by the Cockcroft-Gault formula: eGFR = (140 ± age) 9 weight/72 9 serum creatinine 9 (0.85 if female).

### Animal Experiments

Adult male F344 and Lewis rats (200‐250g) were purchased from Charles River Laboratories (Beijing, China). Animal handling procedures were in accordance with guidelines published by the US National Institutes of Health. All animal experiments were approved by local committee of Soochow University on the care and use of animals.

Kidney transplantation: Orthotopic left kidney transplantation was performed between F344 and Lewis rats as previously described (30). Rats received kidney transplantation were divided into 3 groups. Sham group (Lewis to Lewis), Allo group (F344 to Lewis), Allo+Cur group (F344 to Lewis with the treatment of curcumin). Nephrectomy of the right kidney was performed 10 days after the surgery to evaluate the function of renal allograft. In order to determine the minimum effective dose of curcumin, Allo+Cur group furtherly divided into 3 groups: Curcumin group (100 mg/kg), Curcumin group (200 mg/kg), and Curcumin group (400 mg/kg). Curcumin was suspended in sterile PBS and given once daily by gavage. Cyclosporine A (5 mg/kg bodyweight) was intraperitoneally used to prevent acute rejection for 14 days.

The article "Curcumin Blunts IL-6 Dependent Endothelial‐to‐Mesenchymal Transition to Alleviate Renal Allograft Fibrosis Through Autophagy Activation" was retracted in 2021. Reasons: errors in the data; unreliable images; unreliable results or conclusions.

### Tissue Harvest

According to our previous study, renal allograft fibrosis firstly appeared at 8 weeks after surgery (8). After 8 weeks, 12 weeks, 16weeks of kidney transplantation, allograft tissues were harvested and divided into two parts, which was fixed in paraffin or snap‐frozen in N2 and stored at −80°C.

### Analysis of Cell and Renal Allograft Autophagy

In *vitro* study, cell autophagy was determined by western blot (WB) assays and immunofluorescence (IF). WB was performed to detect the protein abundance of ATG5, ATG7, ATG16L, LC3 I/II, P53 and SQSTM1. Immunofluorescence of LC3II and beclin1was used to evaluate the level of autophagy.

*In vivo* study, we used mRFP-GFP-LC3 adenovirus associated virus (AAV) (32060804, HanBio-Technology; Shanghai, China) to show the kinetics of autophagic flux. AAV was intravenously injected, according to the manufacturer’s instructions. LC3 puncta were examined by fluorescence microscopy (Olympus BX61; Japan). At the same time, autophagy markers were tested by WB assays *via* protein extracted from renal allograft or endothelial cells.

### Cell Culture, Treatment and Transfection

HRGECs and HUVECs were obtained from ScienCell Research Laboratories (4000, 8000, ScienCell; Santiago, USA) and cultured with endothelial cell medium (1001, ScienCell; Santiago, USA), containing 10% FBS (0025, ScienCell; Santiago, USA), 5 ml endothelial cell growth supplement (1052, ScienCell; Santiago, USA) and 5 ml penicillin (10,000 U/ml)/streptomycin (10,000 µg/ml) solution (0503, ScienCell; Santiago, USA). Cells were incubated with IL-6 at indicated time points or different concentrations of IL-6 for 24hours. 3-MA (10 mM) was used as an autophagy inhibitor *in vitro* experiment.

For transfection, HUVECs that were cultured in 6-well plates with non-proliferative medium. The HUVECs were transfected with 25nM of ATG5 siRNA (6345, Cell Signaling Technology; Boston, USA) or control siRNA using Lipofectamine 2000 transfection reagent (11668–019, Invitrogen; California, USA) according to the manufacturer’s instructions.

### Enzyme‐Linked Immunosorbent Assay

The levels of rat serum IL-6 and human cytokine IL-11 were quantified by ELISA kit from MUTISCIENCES (70-EK306/3-96, 70-EK111-96, Beijing, China). Human cytokines (IL-1A, IL-1B, IL-2, IL-4, IL-6, CXCL8, IL-10, TNF-α, TGF-β) were detected with PeliKine Compact human ELISA kit (445804, 437004, 431804, 430301, 430504, 431507, 430604, 430201, 432907, BioLegend; San Diego, USA), according to the manufacturer’s instructions.

### Histopathology

Hematoxylin and eosin and Masson’s trichrome staining were performed as described previously (12). The fibrosis areas were analyzed by Image-Pro Plus 3.0.

The article "Curcumin Blunts IL-6 Dependent Endothelial‐to‐Mesenchymal Transition to Alleviate Renal Allograft Fibrosis Through Autophagy Activation" was retracted in 2021. Reasons: errors in the data; unreliable images; unreliable results or conclusions.

### Immunohistochemistry

Immunohistochemical staining assays were performed to evaluate the expression and distribution of IL-6, fibronectin, α-SMA. Immunohistochemistry staining was performed as described (7). Anti-α-SMA (1:100; Abcam, UK), Anti-IL-6 (1:500; BD, USA), Anti-fibronectin (1:500; BD, USA) antibodies were used as primary antibodies.

### Immunofluorescence

Frozen kidney sections (5μm) and laminin-coated coverslips of HRGECs and HUVECs were used for immunofluorescence. Immunohistochemistry staining was performed as described (31). Primary antibodies used were as followed: Anti-LC3II (1:100; CST, USA), Anti-Beclin1 (1:100; CST, USA), Anti-CD31(1:100; Abcam, UK), Anti-α-SMA (1:100; Abcam, UK), Anti-VE-cadherin (1:100; Abcam, UK).

### Western Blot

Western blot was performed according to the protocol described by Wang et al. by using primary antibodies: Anti-ATG5 (1:1000; CST, USA), Anti-ATG7 (1:1000; CST, USA), Anti-ATG16L (1:1000; CST, USA), Anti-Beclin1 (1:1000; CST, USA), Anti-GAPDH(1:1000; CST, USA), Anti-LC3I-II (1:1000; CST, USA), Anti-P53(1:1000; CST, USA), Anti-SQSTM1(1:1000; CST, USA), Anti-CD31(1:1000; Abcam, UK), Anti-α-SMA (1:1000; Abcam, UK), Anti-VE-cadherin (1:1000; Abcam, UK), Anti-IL-6 (1:5000; Abcam, UK), Anti-fibronectin (1:10000; BD, USA) (31).

### Statistical Analyses

All data were presented as the mean ± SD values determined from three independent experiments. After demonstration of homogeneity of variance with Bartlett test, inter‐group comparisons were made using one‐way analysis of variance (ANOVA). Multiple means were compared using Tukey’s test. The differences between two groups were determined by Student *t* test. Correlation analysis used the Pearson correlation coefficient. A *P* value < 0.05 was considered statistically significant.

## Result

### Autophagy Inactivation Is Associated With EndMT in Patients With CAD

We retrospectively analyzed histologic, cellular, and molecular data from CAD patients and stable control subjects. CAD patients (n=12) had more extensive allograft fibrosis than the stable group (n=10) (**Figures 1A, B**). The number of cells coexpressing the endothelial cell marker CD31 and myofibroblast marker α-SMA (ie, EndMT cells) as detected in biopsy specimens by immunofluorescence analysis was compared between groups. Patients with CAD had significantly more EndMT cells in areas of severe interstitial fibrosis than those in the stable group (**Figures 1C, D**), indicating that EndMT was enhanced in CAD patients.

**Figure 1:** EndMT cells in patients with CAD. Two color immunofluorescence identifies EndMT cells that co-express endothelial cell (CD31, red) and myofibroblast (α-SMA, green) markers in biopsy tissues. **(A)** Representative Masson staining of Stable group (n=10) and CAD (n=12) group. Bar=10 μm. **(B)** Quantification of fibrosis areas in Stable group and CAD group. **(C)** Representative immunofluorescence staining of EndMT cells in Stable group and CAD group. Bar=20 μm. **(D)** Quantification of CD31 and α-SMA co-express cells. LC3 II positive cells in patients with CAD. **(E) **Representative immunofluorescence staining of LC3 II positive cells in Stable group and CAD group. Bar=20 μm. **(F)** Quantification of LC3 II positive cells. Data are mean ± SD. **P<0.01 versus Stable group. **(G)** Correlation analysis of EndMT cells number and area of allograft fibrosis. **(H)** Correlation analysis of number of EndMT cells and allograft function. **(I)** Correlation analysis of numbers of EndMT cells and LC3 II positive cells. **(J)** Correlation analysis of number of LC3 II positive cells and allograft function.

The article "Curcumin Blunts IL-6 Dependent Endothelial‐to‐Mesenchymal Transition to Alleviate Renal Allograft Fibrosis Through Autophagy Activation" was retracted in 2021. Reasons: errors in the data; unreliable images; unreliable results or conclusions.

To examine autophagic flux in greater detail, we examined the expression of microtubule-associated protein 1A/1B-light chain (LC)3-II—one of the main markers of autophagy—by immunofluorescence labeling. The stable group had a higher number of LC3-II–positive cells than CAD patients (**Figures 1E, F**), indicating that autophagy was inactivated in the latter. In patients with CAD, the number of EndMT cells was positively correlated with the area of allograft fibrosis and deterioration of allograft function (**Figures 1G, H**), while the number of LC3-II–positive cells was negatively correlated with the number of EndMT cells and serum creatinine level (**Figures 1I, J**). These findings suggest that autophagy inactivation is associated with EndMT and may contribute to allograft fibrosis.

### Inhibition of Autophagy Promotes EndMT in HUVECs

To confirm the relationship between autophagy inactivation and EndMT, we inhibited autophagy in HUEVCs by 2 methods—namely, small interfering (si)RNA-mediated ATG5 knockdown and 3-methyladenine (3-MA) treatment. HUVECs were transfected with ATG5 siRNA, which resulted in a decrease in the LC3-II/LC3-I ratio and accumulation of sequestosome (SQSTM)1 as well as downregulation of CD31 and VE-cadherin and upregulation of α-SMA (**Figures 2A, B**). A similar effect on HUVECs was observed by pharmacologic inhibition of autophagy with 3-MA (**Figures 2C, D**). Immunofluorescence analysis revealed that the fluorescence intensity of α-SMA was increased whereas that of CD31 and VE-cadherin was decreased by ATG5 knockdown (**Figures 2E, F**). Thus, autophagy inactivation directly contributes to the process of EndMT.

The article "Curcumin Blunts IL-6 Dependent Endothelial‐to‐Mesenchymal Transition to Alleviate Renal Allograft Fibrosis Through Autophagy Activation" was retracted in 2021. Reasons: errors in the data; unreliable images; unreliable results or conclusions.

**Figure 2:** Autophagy inhibition promoted EndMT procession in HUVECs. ATG5 silencing enhanced myofibroblast markers expression and inhibited endothelial cell markers. **(A)** Representative WB of autophagy markers and EndMT markers after si-ATG 5 transfect. **(B)** Quantification of relative protein abundance of autophagy marker (ATG5, LC3 II/I, SQSTM1) and EndMT marker (CD31, VE-cadherin, α-SMA). Data are mean ± SD of five independent experiments. ^*^ *P*<0.05 versus Control siRNA group. 3-MA (10 mM) treatment had the similar effect with ATG5 silencing. **(C)** Representative WB of LC3, SQSTM1, CD31, VE-cadherin and α-SMA. **(D)** Quantification of relative protein abundance of LC3 II/I, SQSTM1, CD31, VE-cadherin and α-SMA. Data are mean ± SD. ^^^ *P*<0.05 versus NS group. **(E)** Representative immunofluorescence staining of ATG5, CD31 and α-SMA indicated the same findings with WB. Bar=20 μm. **(F)** Quantification of relative intensity of ATG5, CD31 and α-SMA. Data are mean ± SD. ^*^ *P*<0.05 versus Control siRNA group.

### EndMT Induced by Autophagy Dysfunction Is Dependent on IL-6

Autophagy defects are associated with the secretion of inflammatory cytokines in many cell types. We investigated the secreted factors responsible for EndMT induced by ATG5 depletion and 3-MA treatment by enzyme-linked immunosorbent assay (ELISA). IL-6 concentration was increased in ATG5 siRNA-transfected HUVECs compared to cells transfected with control siRNA, and in HUVECs treated with 3-MA compared to the normal saline control group (**Figure 3A**). To investigate the mechanism by which IL-6 stimulates EndMT, HUVECs and HRGECs were cultured in the presence of recombinant human IL-6. To determine the appropriate concentration of IL-6 for the *in vivo* experiments, cells were stimulated with different concentrations of IL-6 (0, 1, 10, and 20 ng/ml) for 24 h, and the protein levels of CD31, VE-cadherin, and α-SMA were evaluated by western blotting. We found that treatment with 20 ng/ml IL-6 for 24 h significantly increased the expression of α-SMA and decreased that of CD31 and VE-cadherin **Supplementary Figures 1A, B**. To establish the appropriate IL-6 incubation time, we stimulated HUVECs and HRGECs with 20 ng/ml IL-6 for 0, 6, 12, and 24 h. The results of the western blot analysis showed that EndMT was induced by IL-6 in a time-dependent manner (**Figures 3B–F**). To confirm this observation, cell morphology and CD31 and α-SMA expression levels were examined by immunofluorescence analysis. Morphologic changes in HUVECs from a cobblestone-like to a fibroblast-like appearance were observed after incubation with IL-6 for 24 h (**Figure 3G**); this was accompanied by a decrease in the fluorescence intensity of CD31 and an increase in that of α-SMA (**Figures 3H, I**). Similar results were obtained in HRGECs (**Figures 3J–Q**).

The article "Curcumin Blunts IL-6 Dependent Endothelial‐to‐Mesenchymal Transition to Alleviate Renal Allograft Fibrosis Through Autophagy Activation" was retracted in 2021. Reasons: errors in the data; unreliable images; unreliable results or conclusions.

**Figure 3:** IL-6 incubation promoted phenotype of EndMT in HUVECs and HRGECs. ATG5 silencing and 3-MA treatment enhanced IL-6 secretion of HUVECs. **(A)** Quantification of soluble factors after ATG5 transfection and 3-MA incubation. Data are mean ± SD of five independent experiments. ^+^ *P*<0.05 versus Control siRNA group. ^-^ *P*<0.05 versus NS group. **(B)** Incubation of HUVECs with 20ng/mL IL-6 for the indicated time points. **(C–F)** Quantification of relative protein abundance of FN, CD31, VE-cadherin and α-SMA. Data are mean ± SD of five independent experiments. ^*^ *P*<0.05, ^**^ *P*<0.01 versus IL-6(20ng/ml, 0h) group. **(G)** Representative immunofluorescence staining of CD31 and α-SMA in HUVECs. Bar=20 μm. **(H, I)** Quantification of relative intensity of CD31 and α-SMA in HUVECs. Data are mean ± SD of five independent experiments. ^*^ *P*<0.05, ^**^ *P*<0.01 versus IL-6(20ng/ml, 0h) group. **(J)** Representative immunofluorescence staining of CD31 and α-SMA in HRGECs. Bar=20 μm. **(K–L)** Quantification of relative intensity of CD31 and α-SMA in HRGECs. Data are mean ± SD of five independent experiments. ^*^ *P*<0.05, ^**^ *P*<0.01 versus IL-6(20ng/ml, 0h) group. **(M)** Incubation of HUVECs with 20ng/mL IL-6 for the indicated time points. **(N–Q)** Quantification of relative protein abundance of FN, CD31, VE-cadherin and α-SMA. Data are mean ± SD of five independent experiments. ^*^ *P*<0.05, ^**^ *P*<0.01 versus IL-6(20ng/ml, 0h) group. **(R)** IL-6 nAb alleviated ATG5 siRNA induced EndMT.

To confirm the role of IL-6 in EndMT induced by ATG5 knockdown, we blocked IL-6 using neutralizing antibody. The results of the western blot analysis revealed that in the absence of IL-6, the protein levels of CD31 and VE-cadherin were restored in ATG5-depleted HUVECs and were comparable to those in control siRNA-transfected cells (**Figure 3R**, **Supplementary Figures 2A–D**). Meanwhile, α-SMA expression was reduced by the treatment. These results indicate that EndMT induced by autophagy dysfunction is IL-6–dependent.

### Curcumin Alleviates Allograft Fibrosis, Prevents Functional Deterioration, and Prolongs Survival of Allogeneic Recipients

To determine the appropriate dose of curcumin for *in vivo* experiments, we first treated allogeneic recipient rats with different doses of curcumin. Masson’s trichrome staining revealed that recipient rats treated with 200 and 400 mg/kg curcumin had smaller areas of allograft fibrosis 16 weeks after kidney transplantation compared to rats in the Allo group **Supplementary Figures 3A, B**. Based on this result, a curcumin concentration of 200 mg/kg was used in subsequent experiments. Curcumin alleviated the deterioration of renal function in graft recipients after surgery, which was determined based on blood urea nitrogen and serum creatinine levels, and prolonged the survival of allogeneic recipients (**Figures 4A–C**). Histopathologic analysis revealed that curcumin alleviated fibrosis in the allograft and reduced lumen stenosis (**Figures 4D–F**). Moreover, there was a significant difference in the ratio of α-SMA– and FN-positive areas between the Allo+Cur and Allo groups by immunohistochemistry (**Figures 4D, G, H**).

The article "Curcumin Blunts IL-6 Dependent Endothelial‐to‐Mesenchymal Transition to Alleviate Renal Allograft Fibrosis Through Autophagy Activation" was retracted in 2021. Reasons: errors in the data; unreliable images; unreliable results or conclusions.

**Figure 4:** Curcumin alleviated chronic allograft nephropathy and prolonged survival of allogeneic recipients. **(A, B)** Curcumin protected allograft function deterioration. Data are mean ± SD of five independent experiments. ^*^ *P*<0.05, ^**^ *P*<0.01 *versus* Allo+Cur at indicated times. **(C)** Curcumin prolonged survival of allogeneic recipients. **(D)** Representative H&E, Masson, immunohistochemistry staining of Sham, Allo, Allo+Cur group. Bar=10 μm. **(E–H)** Quantification of allograft fibrosis, vessel stenosis, α-SMA positive cells and FN positive area. Data are mean ± SD of five independent experiments. ^**^ *P*<0.01 *versus* Sham group. ^#^ *P*<0.05, ^##^ *P*<0.01 *versus* Allo group. NS, not significant.

### EndMT Is Attenuated by Curcumin Treatment in a Rat Kidney Transplantation Model

The effect of curcumin on EndMT and allograft fibrosis was examined 12 weeks after surgery by immunohistochemical detection of IL-6 expression. Curcumin treatment markedly reduced the IL-6–positive area (**Figures 5A, B**) and serum IL-6 level in rats at 8, 12, and 16 weeks after kidney transplantation, as determined by ELISA (**Figure 5C**). EndMT in the allograft was assessed by immunofluorescence analysis of CD31 and α-SMA expression (**Figures 5D, E**). Curcumin treatment enhanced the fluorescence intensity of CD31 and reduced that of α-SMA (**Figures 5F, G**). We also calculated the numbers of HUVECs and HRGECs co-expressing CD31 and α-SMA (ie, EndMT cells) and found that they were reduced by curcumin treatment (**Figures 5H, I**), which was supported by the results of the western blot analysis (**Figures 5J, K**).

**Figure 5:** Curcumin alleviated IL-6 dependent EndMT in rat kidney transplant model. **(A)** Representative immunohistochemistry staining of IL-6 in Sham, Allo, Allo+Cur group. Bar=10 μm. **(B)** Quantification of IL-6 positive area. Data are mean ± SD of five independent experiments. ^**^ *P*<0.01 versus Sham group. ^#^ *P*<0.05 versus Allo group. **(C)** Quantification of serum level of IL-6. Data are mean ± SD. ^^^ *P*<0.05, ^^^^ *P*<0.01 versus Allo+Cur group. **(D, E)** Representative immunofluorescence staining of CD31 and α-SMA in Sham group, Allo group and Allo+Cur group. Bar=20 μm. **(F–I)** Quantification of relative intensity of CD31 and α-SMA, Vessel EndMT cells and Glomerular EndMT cells. Data are mean ± SD of five independent experiments. ^*^ *P*<0.05, ^**^ *P*<0.01 versus Sham group. ^#^ *P*<0.05. **(J)** WB assays confirmed our findings. Representative WB image of IL-6, CD31, VE-cadherin, FN and α-SMA. **(K)** Quantification of relative protein abundance of IL-6, CD31, VE-cadherin, FN and α-SMA. Data are mean ± SD of five independent experiments. ^*^ *P*<0.05 *versus* Sham group. ^#^ *P*<0.05 versus Allo group. NS, not significant.

The article "Curcumin Blunts IL-6 Dependent Endothelial‐to‐Mesenchymal Transition to Alleviate Renal Allograft Fibrosis Through Autophagy Activation" was retracted in 2021. Reasons: errors in the data; unreliable images; unreliable results or conclusions.

### Curcumin Induces Autophagy Activation in Renal Allografts

Renal allograft fibrosis progressed over time. At 16 weeks after surgery, the area of renal fibrosis was almost 70% (**Figures 6A, B**), consistent with our previous findings. Activation of autophagy in the grafted kidney was evaluated by western blotting. Autophagic flux in allogeneic recipients was increased compared to the sham group (**Figures 6C**, **Supplementary Figures 4A–C**); the western blot analysis revealed that it peaked at 12 weeks after surgery (**Figure 6C** and **Supplementary Figures 4A–C**). Curcumin treatment increased the number of Beclin1-positive HUVECs and HRGECs in allogeneic recipients (**Figures 6D–G**). We also used GFP-mRFP-LC3 adeno-associated virus to examine autophagic flux. The number of autophagosomes and autolysosomes was increased in allogeneic recipients compared to sham rats (**Figures 6H, I**), and curcumin treatment further increased autophagy activation (**Figures 6H, I**). The results of WB furtherly confirmed our findings (**Figures 6J, K**).

**Figure 6:** Curcumin promoted autophagic flux *in vivo* study. (-): HUVECs without IL-6 incubation. (+): HUVECS with IL-6 incubation. **(A)** Representative Masson staining of Sham and Allo group at indicated time points. Bar=10 μm. **(B)** Quantification of allograft fibrosis. Data are mean ± SD of five independent experiments. ^**^ *P*<0.01, ^##^ *P*<0.01, ^^^^ *P*<0.01 versus Sham group. **(C)** Autophagic flux at indicated time points. Representative WB image of autophagy markers. **(D, E)** Representative immunofluorescence staining of Beclin1 positive cells in Sham group, Allo group and Allo+Cur group. **(D)** Bar=20 μm, **(E)** Bar=15 μm. **(F, G)** Quantification of Beclin1 positive vessel endothelial cells and glomerular endothelial cells. ^*^ *P*<0.05, ^**^ *P*<0.01 versus Sham group. ^#^ *P*<0.05 versus Allo group. **(H)** Representative immunofluorescence staining of GFP-mRFP-LC3. Bar=20 μm. **(I)** Quantification of autophagosomes and autolysosomes. Data are mean ± SD of five independent experiments. Autophagosomes: ^a^ *P*<0.05 versus Sham group. ^b^ *P*>0.05 versus Allo group. Autolysosomes: ^c^ *P*<0.05 versus Sham group. ^d^ *P*>0.05 versus Allo group. **(J)** Findings of WB confirmed our immunofluorescence results. **(K)** Quantification of relative protein abundance of autophagy marker. Data are mean ± SD of five independent experiments. ^*^ *P*<0.05 versus Sham group. ^#^ *P*<0.05 *versus* Allo group.

The article "Curcumin Blunts IL-6 Dependent Endothelial‐to‐Mesenchymal Transition to Alleviate Renal Allograft Fibrosis Through Autophagy Activation" was retracted in 2021. Reasons: errors in the data; unreliable images; unreliable results or conclusions.

### Curcumin Inhibits IL-6–Dependent EndMT by Promoting Autophagy Activation in HUVECs

To confirm our vivo findings, we evaluated the effect of curcumin on IL-6–dependent EndMT. We first determined the effective therapeutic concentration of curcumin for *in vitro* experiments and found that 10, 30, and 50 μM curcumin reversed IL-6–dependent EndMT and promoted autophagy using EGFP-conjugated LC3-II to visualize autophagic flux in HUVECs (**Figures 7A, B**). These results were confirmed by western blotting (**Figures 7B, C**) and immunofluorescence analysis (**Figures 7D–F**). Thus, curcumin blocks IL-6–dependent EndMT to alleviate renal allograft fibrosis *via* autophagy induction (**Figure 7G**). A model is proposed to illustrate the fibrotic mechanism involved in EndMT induced by IL-6 in the pathogenesis of allogeneic kidney interstitial fibrosis and the therapeutic mechanism of Curcumin (**Figure 7H**).

**Figure 7:** Curcumin attenuated IL-6 dependent EndMT *via* autophagy activation. (-): HUVECs without IL-6 incubation. (+): HUVECS with IL-6 incubation. **(A)** Representative WB of autophagy markers and EndMT markers. **(B)** Quantification of protein abundance of autophagy markers and EndMT markers. Data are mean ± SD. ^*^ *P*<0.05 versus IL-6 20ng/ml+Cur 0μm group. ^^^ *P*<0.05 *versus* IL-6 0ng/ml+Cur 0μm group. **(C)** Representative immunofluorescence staining of LC3 II in HUVECs. Bar=20 μm. **(D)** Quantification of average number of LC3 II puncta. Data are mean ± SD of five independent experiments. ^++^ *P*<0.01 *versus* IL-6 20ng/ml+Cur 10μm group. ^##^ *P*<0.01 versus IL-6 20ng/ml+Cur 50μm group. **(E)** Curcumin inhibited HUVECs transition to EndMT phenotype. Representative immunofluorescence staining of CD31 and α-SMA in HUVECs. Bar=20 μm. **(F, G)** Quantification of relative intensity of CD31 and α-SMA. Data are mean ± SD of five independent experiments. ^*^ *P*<0.05 *versus* IL-6 20ng/ml+Cur 10μm group. ^#^ *P*<0.05 *versus* IL-6 20ng/ml+Cur 50μm group. **(H)** A model is proposed to illustrate the fibrotic mechanism involved in EndMT induced by IL-6 in the pathogenesis of allogeneic kidney interstitial fibrosis and the therapeutic mechanism of Curcumin. NS, not significant.

The article "Curcumin Blunts IL-6 Dependent Endothelial‐to‐Mesenchymal Transition to Alleviate Renal Allograft Fibrosis Through Autophagy Activation" was retracted in 2021. Reasons: errors in the data; unreliable images; unreliable results or conclusions.

## Discussion

Autophagy is critical for homeostasis in cells and tissues (32, 33); however, the role of autophagy in the development of renal allograft fibrosis is unknown. This was investigated in the present study using *in vitro* and *in vivo* models as well as clinical specimens. Our findings were as follows. 1) Autophagy inactivation was associated with EndMT in CAD patients. 2) Inhibition of autophagy induced EndMT *in vitro*. 3) EndMT induced by defective autophagy was IL-6–dependent. 4) Curcumin attenuated renal allograft fibrosis *in vivo*. 5) Curcumin inhibited IL-6–dependent EndMT by inducing autophagy *in vitro* and *in vivo*.

Transforming growth factor (TGF)-β1 is a well-known inducer of EndMT and was shown to be involved in the development of renal allograft fibrosis (31); TGF-β signaling has also been linked to both EndMT induction and autophagy (34–36). We initially hypothesized that activation of TGF-β signaling was responsible for EndMT induction in autophagy-deficient endothelial cells; however, we did not observe increased secretion of TGF-β after ATG5 knockdown. TGF-β neutralization and inhibition of Mothers against decapentaplegic homolog (SMAD)3 phosphorylation did not suppress EndMT induced by ATG5 depletion in HMVECs, although TGF-β secretion was increased (29). In order to identify the cytokines responsible for knockdown-induced EndMT, we analyzed changes in the levels of soluble factors by ELISA and found that IL-6 level was increased in HUVECs in the absence of ATG5. IL-6 application induced an EndMT phenotype in HUVECs and HRGECs, and EndMT induced by ATG5 depletion was rescued by IL-6 neutralizing antibody treatment. Similar results were observed in our *in vivo* experiments. This is the first study demonstrating the induction of EndMT by IL-6 in renal allografts.

Autophagy is known to be involved in the regulation of EndMT (37, 38). Based on our finding that defective autophagy was associated with EndMT in CAD patients, we speculated that autophagy plays a protective role in allograft fibrosis. In our rat kidney transplantation model, autophagy was markedly increased in the Allo group compared to the sham group; curcumin increased the expression of autophagy-related proteins and attenuated EndMT, which was consistent with our *in vitro* results. Thus, in contrast to the finding that inhibition of autophagy prolonged recipient survival in a rat liver transplantation model (23), autophagy prevents allograft fibrosis following kidney transplantation. Our study provides the first evidence of the protective effect of curcumin against allograft EndMT, and indicates that therapeutic strategies targeting autophagy can prevent renal allograft fibrosis.

The article "Curcumin Blunts IL-6 Dependent Endothelial‐to‐Mesenchymal Transition to Alleviate Renal Allograft Fibrosis Through Autophagy Activation" was retracted in 2021. Reasons: errors in the data; unreliable images; unreliable results or conclusions.

In our study, IL-6 synthesis and secretion were induced by autophagy inactivation in endothelial cells; however, IL-6 application had no effect on autophagy induction (**Supplementary Figure 5**). The contribution of autophagy to cytokine synthesis and secretion varies according to the cell type. In breast epithelial cells, autophagy inactivation enhanced IL-6 secretion but not synthesis, which was associated with an invasive type of RAS-transformed breast epithelial cells (39). On the other hand, autophagy inactivation induced IL-6 synthesis but not secretion in fibroblasts, which was associated with cell senescence (40, 41). These variable effects of autophagy on cytokines reflect the diverse physiologic or pathologic settings. Autophagy in endothelial cells is an important regulator of redox homeostasis (42). Reactive oxygen species (ROS) were shown to increase IL-6 secretion by endothelial cells, which is a potential mechanism by which autophagy inactivation induces EndMT. Myeloperoxidase (MPO) level represents the degree of tissue damage caused by ROS, while superoxide dismutase (SOD) level reflects the cell’s ability to scavenge ROS. In our study, ATG5 knockdown increased MPO and decreased SOD levels in endothelial cells in the Allo group compared to the sham group (**Supplementary Figure 6**), suggesting that ROS stimulated the production and release of IL-6, leading to EndMT in the absence of autophagy. Conversely, induction of autophagy may reduce IL-6 production by inhibiting ROS production. Additional studies are needed to examine these possibilities.

In conclusion, we demonstrated that curcumin alleviated renal allograft fibrosis in rats and inhibited EndMT, possibly by stimulating autophagy. These results indicate that curcumin is an effective natural alternative to conventional drugs for the treatment of allograft fibrosis and can improve the clinical outcome of patients undergoing kidney transplantation.

## Data Availability Statement

The raw data supporting the conclusions of this article will be made available by the authors, without undue reservation.

## Ethics Statement

The studies involving human participants were reviewed and approved by Human Ethics Committee of Soochow University. The patients/participants provided their written informed consent to participate in this study. The animal study was reviewed and approved by Animal Ethics Committee of Soochow University. Written informed consent was obtained from the individual(s) for the publication of any potentially identifiable images or data included in this article.

The article "Curcumin Blunts IL-6 Dependent Endothelial‐to‐Mesenchymal Transition to Alleviate Renal Allograft Fibrosis Through Autophagy Activation" was retracted in 2021. Reasons: errors in the data; unreliable images; unreliable results or conclusions.

## Author Contributions

Study design: DW. Data collection: JZ and MY. Software material: MZ. Data analysis: QK, ML, and BW. Manuscript preparation: JZ, MY, and MZ. All authors contributed to the article and approved the submitted version.

## Funding

This work was supported by the Science Project of Changzhou Science and Technology Bureau (CJ20190064).

## Conflict of Interest

The authors declare that the research was conducted in the absence of any commercial or financial relationships that could be construed as a potential conflict of interest.

## References

[1] ChapmanJR. What Are the Key Challenges We Face in Kidney Transplantation Today? Transplant Res (2013) 2(Suppl 1):S1. 10.1186/2047-1440-2-s1-s1 24565161PMC3834535

[2] BalujaPHaragsimLLaszikZ. Chronic Allograft Nephropathy. Adv Chronic Kidney Dis (2006) 13(1):56–61. 10.1053/j.ackd.2005.11.004 16412971

[3] FadiliWHabib AllahMLaouadI. Chronic Renal Allograft Dysfunction: Risk Factors, Immunology and Prevention. Arab J Nephrol Transplant (2013) 6(1):45–50.23282234

[4] CostaJSAlvesRSousaVMarinhoCRomãozinhoCSantosL. Fibrogenesis in Kidney Transplant: Dysfunction Progress Biomarkers. Transplant Proc (2017) 49(4):787–91. 10.1016/j.transproceed.2017.01.063 28457395

[5] VanhoveTGoldschmedingRKuypersD. Kidney Fibrosis: Origins and Interventions. Transplantation (2017) 101(4):713–26. 10.1097/tp.0000000000001608 PMC722859327941433

[6] XuZZhaoCWangZTaoJHanZZhangW. Interleukin-33 Levels Are Elevated in Chronic Allograft Dysfunction of Kidney Transplant Recipients and Promotes Epithelial to Mesenchymal Transition of Human Kidney (HK-2) Cells. Gene (2018) 644:113–21. 10.1016/j.gene.2017.11.010 29122645

[7] ZhaoCXuZWangZSuoCTaoJHanZ. Role of Tumor Necrosis Factor-α in Epithelial-to-Mesenchymal Transition in Transplanted Kidney Cells in Recipients With Chronic Allograft Dysfunction. Gene (2018) 642:483–90. 10.1016/j.gene.2017.11.059 29174387

[8] ZhouJChengHWangZChenHSuoCZhangH. Bortezomib Attenuates Renal Interstitial Fibrosis in Kidney Transplantation Via Regulating the EMT Induced by TNF-α-Smurf1-Akt-mTOR-P70S6K Pathway. J Cell Mol Med (2019) 23(8):5390–402. 10.1111/jcmm.14420 PMC665343531140729

[9] WangYYJiangHPanJHuangXRWangYCHuangHF. Macrophage-to-Myofibroblast Transition Contributes to Interstitial Fibrosis in Chronic Renal Allograft Injury. J Am Soc Nephrol (2017) 28(7):2053–67. 10.1681/asn.2016050573 PMC549127828209809

[10] ZeisbergEMTarnavskiOZeisbergMDorfmanALMcMullenJRGustafssonE. Endothelial-to-Mesenchymal Transition Contributes to Cardiac Fibrosis. Nat Med (2007) 13(8):952–61. 10.1038/nm1613 17660828

The article "Curcumin Blunts IL-6 Dependent Endothelial‐to‐Mesenchymal Transition to Alleviate Renal Allograft Fibrosis Through Autophagy Activation" was retracted in 2021. Reasons: errors in the data; unreliable images; unreliable results or conclusions.

[11] LiJLiCZhuangQPengBZhuYYeQ. The Evolving Roles of Macrophages in Organ Transplantation. J Immunol Res (2019) 2019:5763430. 10.1155/2019/5763430 31179346PMC6507224

[12] WangZHanZTaoJWangJLiuXZhouW. Transforming Growth Factor-β1 Induces Endothelial-to-Mesenchymal Transition Via Akt Signaling Pathway in Renal Transplant Recipients With Chronic Allograft Dysfunction. Ann Transplant (2016) 21:775–83. 10.12659/aot.899931 27994216

[13] GloverEKJordanNSheerinNSAliS. Regulation of Endothelial-to-Mesenchymal Transition by MicroRNAs in Chronic Allograft Dysfunction. Transplantation (2019) 103(4):e64–73. 10.1097/tp.0000000000002589 PMC643672730907855

[14] GlickDBarthSMacleodKF. Autophagy: Cellular and Molecular Mechanisms. J Pathol (2010) 221(1):3–12. 10.1002/path.2697 20225336PMC2990190

[15] MizushimaNKomatsuM. Autophagy: Renovation of Cells and Tissues. Cell (2011) 147(4):728–41. 10.1016/j.cell.2011.10.026 22078875

[16] ZhaoXCLivingstonMJLiangXLDongZ. Cell Apoptosis and Autophagy in Renal Fibrosis. Adv Exp Med Biol (2019) 1165:557–84. 10.1007/978-981-13-8871-2_28 31399985

[17] LuCYangYZhuYLvSZhangJ. An Intervention Target for Myocardial Fibrosis: Autophagy. BioMed Res Int (2018) 2018:6215916. 10.1155/2018/6215916 29850542PMC5911341

[18] Cosin-RogerJCanetFMacias-CejaDCGisbert-FerrándizLOrtiz-MasiáDEspluguesJV. Autophagy Stimulation as a Potential Strategy Against Intestinal Fibrosis. Cells (2019) 8(9):1078. 10.3390/cells8091078 PMC677011831540207

[19] ZouJLiuYLiBZhengZKeXHaoY. Autophagy Attenuates Endothelial-to-Mesenchymal Transition by Promoting Snail Degradation in Human Cardiac Microvascular Endothelial Cells. Biosci Rep (2017) 37(5):BSR20171049. 10.1042/bsr20171049 28811357PMC5587916

[20] WangYRijalBXuMLiZAnYZhangF. Renal Denervation Improves Vascular Endothelial Dysfunction by Inducing Autophagy Via AMPK/mTOR Signaling Activation in a Rat Model of Type 2 Diabetes Mellitus With Insulin Resistance. Acta Diabetol (2020) 57(10):1227–43. 10.1007/s00592-020-01532-6 32488498

[21] LiangXZhangTShiLKangCWanJZhouY. Ampelopsin Protects Endothelial Cells From Hyperglycemia-Induced Oxidative Damage by Inducing Autophagy Via the AMPK Signaling Pathway. Biofactors (2015) 41(6):463–75. 10.1002/biof.1248 26644014

[22] XiongADuanLChenJFanZZhengFTanZ. Flt3L Combined With Rapamycin Promotes Cardiac Allograft Tolerance by Inducing Regulatory Dendritic Cells and Allograft Autophagy in Mice. PloS One (2012) 7(10):e46230. 10.1371/journal.pone.0046230 23056267PMC3462742

[23] ChenXWangLDengYLiXLiGZhouJ. Inhibition of Autophagy Prolongs Recipient Survival Through Promoting CD8(+) T Cell Apoptosis in a Rat Liver Transplantation Model. Front Immunol (2019) 10:1356. 10.3389/fimmu.2019.01356 31258533PMC6587890

The article "Curcumin Blunts IL-6 Dependent Endothelial‐to‐Mesenchymal Transition to Alleviate Renal Allograft Fibrosis Through Autophagy Activation" was retracted in 2021. Reasons: errors in the data; unreliable images; unreliable results or conclusions.

[24] SunXLiuYLiCWangXZhuRLiuC. Recent Advances of Curcumin in the Prevention and Treatment of Renal Fibrosis. BioMed Res Int (2017) 2017:2418671. 10.1155/2017/2418671 28546962PMC5435901

[25] YuYSunJWangRLiuJWangPWangC. Curcumin Management of Myocardial Fibrosis and Its Mechanisms of Action: A Review. Am J Chin Med (2019) 47(8):1675–710. 10.1142/s0192415x19500861 31786946

[26] WuCQiuYBSunXQChenDWuYXPangQF. [Effects of Curcumin on Liver Fibrosis Induced by Cholestasis in Mice]. Zhongguo Ying Yong Sheng Li Xue Za Zhi (2019) 35(5):468–72. 10.12047/j.cjap.5796.2019.102 31894682

[27] AnandPKunnumakkaraABNewmanRAAggarwalBB. Bioavailability of Curcumin: Problems and Promises. Mol Pharm (2007) 4(6):807–18. 10.1021/mp700113r 17999464

[28] KongDZhangZChenLHuangWZhangFWangL. Curcumin Blunts Epithelial-Mesenchymal Transition of Hepatocytes to Alleviate Hepatic Fibrosis Through Regulating Oxidative Stress and Autophagy. Redox Biol (2020) 36:101600. 10.1016/j.redox.2020.101600 32526690PMC7287144

[29] TakagakiYLeeSMDongqingZKitadaMKanasakiKKoyaD. Endothelial Autophagy Inactivation Induces IL6 - Dependent Endothelial Mesenchymal Transition and Organ Fibrosis. Autophagy (2020) 16(10):1905–14. 10.1080/15548627.2020.1713641 PMC838662231965901

[30] VogelbacherRMeisterSGückelEStarkeCWittmannSStiefA. Bortezomib and Sirolimus Inhibit the Chronic Active Antibody-Mediated Rejection in Experimental Renal Transplantation in the Rat. Nephrol Dial Transplant (2010) 25(11):3764–73. 10.1093/ndt/gfq230 20466656

[31] WangZHanZTaoJWangJLiuXZhouW. Role of Endothelial-to-Mesenchymal Transition Induced by TGF-β1 in Transplant Kidney Interstitial Fibrosis. J Cell Mol Med (2017) 21(10):2359–69. 10.1111/jcmm.13157 PMC561868028374926

[32] LevineBKroemerG. Autophagy in the Pathogenesis of Disease. Cell (2008) 132(1):27–42. 10.1016/j.cell.2007.12.018 18191218PMC2696814

[33] LevineBKroemerG. Biological Functions of Autophagy Genes: A Disease Perspective. Cell (2019) 176(1-2):11–42. 10.1016/j.cell.2018.09.048 30633901PMC6347410

[34] ZhangCZhangXXuRHuangBChenAJLiC. TGF-β2 Initiates Autophagy Via Smad and Non-Smad Pathway to Promote Glioma Cells’ Invasion. J Exp Clin Cancer Res (2017) 36(1):162. 10.1186/s13046-017-0628-8 29145888PMC5689187

[35] MaoXXuZXuXZengMZhaoZZhangZ. TGF-β1 Inhibits the Autophagy of Podocytes by Activating mTORC1 in IgA Nephropathy. Exp Cell Res (2019) 385(1):111670. 10.1016/j.yexcr.2019.111670 31600491

[36] CooleyBCNevadoJMelladJYangDSt HilaireCNegroA. TGF-β Signaling Mediates Endothelial-to-Mesenchymal Transition (EndMT) During Vein Graft Remodeling. Sci Transl Med (2014) 6(227):227ra34. 10.1126/scitranslmed.3006927 PMC418140924622514

The article "Curcumin Blunts IL-6 Dependent Endothelial‐to‐Mesenchymal Transition to Alleviate Renal Allograft Fibrosis Through Autophagy Activation" was retracted in 2021. Reasons: errors in the data; unreliable images; unreliable results or conclusions.

[37] ZhangRHuangXQJiangYYLiNWangJChenSY. LncRNA TUG1 Regulates Autophagy-Mediated Endothelial-Mesenchymal Transition of Liver Sinusoidal Endothelial Cells by Sponging miR-142-3p. Am J Transl Res (2020) 12(3):758–72.PMC713707032269710

[38] LiZLiXZhuYChenQLiBZhangF. Protective Effects of Acetylcholine on Hypoxia-Induced Endothelial-to-Mesenchymal Transition in Human Cardiac Microvascular Endothelial Cells. Mol Cell Biochem (2020) 473(1–2):101–10. 10.1007/s11010-020-03811-w 32602017

[39] LockRKenificCMLeidalAMSalasEDebnathJ. Autophagy-Dependent Production of Secreted Factors Facilitates Oncogenic RAS-Driven Invasion. Cancer Discov (2014) 4(4):466–79. 10.1158/2159-8290.Cd-13-0841 PMC398000224513958

[40] NaritaMYoungARArakawaSSamarajiwaSANakashimaTYoshidaS. Spatial Coupling of mTOR and Autophagy Augments Secretory Phenotypes. Science (2011) 332(6032):966–70. 10.1126/science.1205407 PMC342629021512002

[41] YoungARNaritaMFerreiraMKirschnerKSadaieMDarotJF. Autophagy Mediates the Mitotic Senescence Transition. Genes Dev (2009) 23(7):798–803. 10.1101/gad.519709 19279323PMC2666340

[42] AliMHSchlidtSAChandelNSHynesKLSchumackerPTGewertzBL. Endothelial Permeability and IL-6 Production During Hypoxia: Role of ROS in Signal Transduction. Am J Physiol (1999) 277(5):L1057–65. 10.1152/ajplung.1999.277.5.L1057 10564193

